The article "The Pharmacological Mechanism of Xiyanping Injection for the Treatment of Novel Coronavirus Pneumonia (COVID-19): Based on Network Pharmacology Strategy" was published in 2022. Journal: Evid Based Complement Alternat Med.

# The Pharmacological Mechanism of Xiyanping Injection for the Treatment of Novel Coronavirus Pneumonia (COVID-19): Based on Network Pharmacology Strategy

**DOI:** 10.1155/2022/9152201

**Published:** 2022-07-08

**Authors:** Liang-jing Xia, Liang-ming Zhang, Kun Yang, Tong Chen, Xian-wen Ye, Zi-jun Yan

**Affiliations:** ^1^Department of Pharmacy, Panzhihua Central Hospital, Panzhihua 617067, China; ^2^School of Pharmacy and Pharmaceutical Sciences (Institute of Pharmaceutical Sciences), Shandong First Medical University (Shandong Academy of Medical Sciences), Jinan 250117, China; ^3^School of Pharmacy, Dali University, Dali 671000, China; ^4^School of Pharmaceutical Sciences and Yunnan Key Laboratory of Pharmacology for Natural Products, Kunming Medical University, Kunming 650500, China; ^5^Centre of TCM Processing Research, Beijing University of Chinese Medicine, Beijing 102488, China

## Abstract

**Purpose:**

The possible mechanism of Xiyanping injection treatment COVID-19 is discussed through the network pharmacology.

**Methods:**

Obtaining the chemical structure of Xiyanping injection through the patent application and obtaining control compounds I, II, III, IV, V, Yanhuning injection (VI, VII), Chuanhuning injection (VIII, IX), 10 compounds were analyzed by D3Targets-2019-nCoV. The human anti-COVID-19 gene in COVID-19 DisGeNET was intersected with the CTD Andrographolide target gene and then combined with D3Targets-2019-nCoV, resulting in 93 genes, using the Venny 2.1 platform. The PPI network was constructed by the String platform and Cytoscape 3.8.2 platform. The GO, KEGG, and tissue of the target were analyzed using the Metascape platform and DAVID platform. The gene expression in the respiratory system was analyzed using the ePlant platform. The CB-Dock is used for the docking verification and degree values of the first 20 genes.

**Results:**

Finally, 1599 GO and 291 KEGG results were obtained. GO is mostly associated with the cell stress response to chemicals, the cell response to oxidative stress, and the cell response to reactive oxygen species. In total, 218 KEGG pathway concentrations were related to infection and other diseases and 73 signaling pathways mostly related to inflammation and immune pathways, such as TNF signaling pathway and MAPK signaling pathway. The molecular docking results show that Xiyanping injection, compound III, has a good docking relationship with 20 target proteins such as HSP90AA1. Tissue has 22 genes that are pooled in the lungs.

**Conclusion:**

Xiyanping injection may inhibit the release of various inflammatory factors by inhibiting intracellular pathways such as MAPK and TNF. It acts on protein targets such as HSP90AA1 and plays a potential therapeutic role in COVID-19. Thus, compound III may be treated as a potential new drug for the treatment of COVID-19 and the Xiyanping injection may treat patients with COVID-19 infection.

The article "The Pharmacological Mechanism of Xiyanping Injection for the Treatment of Novel Coronavirus Pneumonia (COVID-19): Based on Network Pharmacology Strategy" was published in 2022. Journal: Evid Based Complement Alternat Med.

## 1. Introduction

According to expert consensus, Xiyanping injection belongs to Chinese medicine injections, primarily composed of *sodium((1R, 2R, 4aR, 8aS)-2-hydroxy-5-((E)-2-((S)-4-hydroxy-2-oxodihydrofuran-3(2H)- ylidene) ethyl)-1,4a,6-trimethyl-1,2,3,4,4a,7,8,8a-octahydronaphthalen-1-yl)methyl sulfate* (C_20_H_29_O_5_·SO_3_Na). It mainly has anti-inflammatory, antibacterial, anticough, and other effects and enhances the body's immunity, [1]. In the “2019 Novel Coronavirus Diagnosis and Treatment Program” (Trial 6th Edition) implemented by the State Health and Construction Commission of China, the virus infection is heavy and critical or combined with mild bacterial infection, and the treatment of Xiyanping injection is recommended with Chinese medicine injection. The recommended usage is as follows: 0.9% sodium chloride injection 250 mL plus Xiyanping injection 100 mg b.i.d. [2]. The drug has been on the market for more than 30 years. In 2016, Xiyanping injection ranked in the top three in the market for Chinese medicine injections in the clear-heat detoxification category, with market size of about 2.6 billion yuan, often used in pediatrics [3].

Coronaviruses (CoVs) consist of a single positive-chain RNA virus that belongs to the coronavirus group and can develop into respiratory, intestinal, nervous, reproductive, and other diseases in infected animals and humans [4]. In 2019, some hospitals in Wuhan City, Hubei Province, have found several cases of unexplained pneumonia with a history of exposure to the South China seafood market, which has been confirmed as a new type of coronavirus infection caused by acute respiratory infections. The World Health Organization has named the virus “COVID-19” [5]. Similar to the pathological mechanism of Severe Acute Respiratory Syndrome (SARS), SARS-CoV-2 infections disrupt the epithelial-endothelial barrier in the bronchial and alveoli, causing alveoli-capillary oxygen transfer dysfunction and impaired oxygen diffusion. In patients with severe COVID-19, severe coagulation dysfunction and thrombosis and sepsis further lead to multiple organ failures [6]. Zhong Nanshan's team reported in the literature that 63.4% of COVID-19 patients had a fever and lung abnormalities in chest CT scans; experimental studies have shown that patients with COVID-19 have lymphocyte reduction and increased levels of reactive protein (CRP) [7].

Recently, network pharmacology has been widely used in the study of Chinese medicine anti-SARS-CoV-2 [8]. The emerging network pharmacology technology can be widely used to explore the possible mechanism of Chinese medicine to treat diseases through multicomponent, multitarget, and multichannel levels and to explore potential therapeutic drugs [9]. The Chinese medicine injections in the New Coronary Virus Pneumonia Treatment Programme (Trial 7) [10] are included in the recommended SARS-CoV-2 treatment options, such as Xiyanping injection, Xuebijing injection, Reduning, Tanreqing injection, Xingnaoling injection, Shenfu injection, Shenmai injection, and Shengmai injection. This has also raised awareness and acceptance of Chinese medicine injections. In Wuhan Jinyintan Hospital, Wuhan Lung Hospital, Huazhong University of Science, and Technology Tongji Medical College affiliated Concord Hospital, seriously ill patients by the Chinese and Western Medical Federation, more patients used Chinese medicine injections, achieved good results. Professor Zhangboli said “for patients with mild illness, a large number of practices have proved that Chinese medicine can improve symptoms, shorten the course of treatment, and promote healing” [11]. Mild patients often present with fever, dry cough, and fatigue symptoms mainly. Some patients have wheezing, and lungs scattered in the oozing symptoms; Chinese medicine has detoxification, cough relief, and other good therapeutic effects. He led the clinical study of the Wuhan Fire Line project. The phase analysis shows that the first batch of 52 patients in Hubei Province combined with Western medicine hospital clinical control study: including 34 cases of Chinese and Western medicine combined treatment group, 18 cases of the simple Western medicine treatment group. The data analysis results show that compared with the Western medicine group, the clinical symptoms of the combination group of Chinese and Western medicine were shortened by 2 days. The normal temperature was reduced by 1.7 days. The average number of hospital days was shortened by 2.2 days. The CT image improvement rate was increased by 22%, and the clinical cure rate was increased by 33% [11].

The article "The Pharmacological Mechanism of Xiyanping Injection for the Treatment of Novel Coronavirus Pneumonia (COVID-19): Based on Network Pharmacology Strategy" was published in 2022. Journal: Evid Based Complement Alternat Med.

Based on clinical data, this article uses network pharmacology to explore the possible mechanism of Xiyanping injection anti-SARS-CoV-2, while andrographolide, compound III, can be used as a potential new anti-SARS-CoV-2 drug (Figure 1).

## 2. Materials and Methods

### 2.1. Collection of Target Compounds

We obtained the chemical structures of six andrographolide salts, including Xiyanping injection and other andrographolide salts synthesized in process production, through the contents in the patent book of pharmaceutical companies. These five compounds were derived from the production process of Xiyanping injection, but they were not produced in the market as the objects of subsequent pharmacodynamic development, and there were no related clinical studies: I, II, III, IV, and V. We obtained similar andrographolide Chinese medicine injections via the DrugBank [12] platform (https://go.drugbank.com/): Yanhuning injection compounds: VI and VII; Chuanhuning injection compounds: VIII and IX. Ten compounds are drawn and saved in SDF format via ChemDraw 20.0 software [13].

### 2.2. Screening of Disease Targets

Based on the D3Targets-2019-nCoV platform [14] (https://www.d3pharma.com/D3Targets-2019-nCoV/index.php), the Xiyanping injection anti-COVID-19-related target genes were docked. We obtained human gene targets related to andrographolide based on the CTD platform [15] (https://ctdbase.org/). The CTD platform [15]captures the set of genetic targets that andrographolide acts on in humans; the Human anti-COVID-19 gene dataset on the COVID-19 DisGeNET platform [16] (https://ctdbase.org/) takes the target intersection collection of these two gene sets through the Venny 2.1 platform (https://bioinfogp.cnb.csic.es/tools/venny/). The collection is then merged with the human anti-COVID-19 target obtained by the D3Targets-2019-nCoV platform [14]. Finally, a target set of the andrographolide drug Xiyanping injection anti-COVID-19 was obtained [(CTD ∩ COVID-19 DisGeNET)∪D3Targets-2019-nCoV]−[(CTD ∩ COVID-19 DisGeNET)∩ D3Targets-2019-nCoV].

### 2.3. Target Gene Network Construction and Analysis

The target protein is converted into the corresponding gene name through the UniProt platform [17] (https://www.uniprot.org/), and the target protein interaction network (PPI network) is built through the String platform [18] (https://www.string-db.org/). Finally, a compound-target PPI network is built using the Cytoscape 3.8.2 software platform [19].

### 2.4. GO and KEGG Pathway Enrichment Analysis

To further analyze the function of the target, the target is uploaded to the Metascape platform [20] (https://metascape.org/); the species is limited to “*H. sapiens*,” the threshold *P* < 0.05, and its GO biofunction (biological process (BP), molecular function (MF), and cell composition (CC)) enrichment analysis is carried out. At the same time, KEGG signal path enrichment analysis and tissue structural analyses are carried out through the DAVID platform [21] (https://david.ncifcrf.gov/), and Enrichment Plot is drawn through the image GP platform (http://www.ehbio.com/).

### 2.5. Drug Ingredients: Protein Targets' Molecular Docking

Download the Human Target Protein (Table 1) in the Top 20 Degrees from the PDB platform [22] (https://www.rcsb.org/): 20 target macromolecules, hydrogenation, removal of water molecules, removal of ligands, etc., through Discovery Studio 2019 Client software [23]. The target component and macromolecules are uploaded to the CB-Dock platform [24] (https://clab.labshare.cn/cb-dock/php/) for molecular docking to bind the energy ≤ −5.0 kcal/mol as the basis for molecular-target interactions [25]. The docking results are mapped to heatmap via the image GP platform, and the binding sites and patterns of ligand drugs and target proteins are observed through Discovery Studio 2019 Client software [23].

The article "The Pharmacological Mechanism of Xiyanping Injection for the Treatment of Novel Coronavirus Pneumonia (COVID-19): Based on Network Pharmacology Strategy" was published in 2022. Journal: Evid Based Complement Alternat Med.

### 2.6. Organizing Enrichment Analysis

We performed organizational analysis via the DAVID platform [21], analysis of Xiyanping injection Vina scores of higher HSP90AA1, CAT gene target and compound III Vina score of higher TNF, and FOS gene target and observed the relationship between genes and tissues, using the Human eFP Browser platform [26].

## 3. Results

### 3.1. Screening of Active Compounds

We obtained the chemical structure of andrographolide-sulfonate: Xiyanping injection, I, II, III, IV, and V through a patent application for Jiangxi Qingfeng Pharmaceuticals [27]. The DrugBank Platform has similar andrographolide Chinese injections: Yanhuning injection compounds: VI and VII; Chuanhuning injection compounds: VIII and IX (Figure 2).

### 3.2. Target Gene Network Analysis

D3Targets-2019-nCoV platform database [14] was used to collect 34 human genes. The 1812 human genes associated with COVID-19 in the DisGeNET platform [16] were intersected with 150 *Homo sapiens* target genes in the CTD platform [15]. For andrographolide, 60 genes (Figure 3) were collected through the Venny 2.1 platform. The genetic results of the D3Targets-2019-nCoV platform [14] were combined to obtain 93 genes (Table 1, Figure 4). We standardized the 93 target genes obtained with the UniProt platform [17]. By analyzing 93 genes through the String platform [18], the number of nodes of the network graph was 93, 1174 edges, and the PPI rich *P*-value: <1.0*e* − 16, which is considered to have strong biological significance. The target PPI network was built using the Cytoscape 3.8.2 platform [19], in which 89 gene nodes were associated, average degree value of 26.38. The circle is the target gene, and the base color with the degree value less than the average value is yellow, and the larger the degree value is, the closer it is to green and the larger the shape is (Figure 5). The top 20 degree values in the PPI network diagram are used as the core targets, in which 20 targets, such as target AKT1 (Degree: 75.0), TP53 (Degree: 65.0), and TNF (Degree: 64.0), are all greater than the average of 1.5 times. These targets are considered to be the main target points for the anti-COVID-19 by the andrographolide drugs (Table 2).

The article "The Pharmacological Mechanism of Xiyanping Injection for the Treatment of Novel Coronavirus Pneumonia (COVID-19): Based on Network Pharmacology Strategy" was published in 2022. Journal: Evid Based Complement Alternat Med.

### 3.3. GO and KEGG Signal Path Enrichment Analysis

GO Enrichment 2343 items through the Metascape platform, which can be clustered into five items by their target properties (Figure 6). The most significant category of items is the mitogen-activated protein kinase MAPK family (MAPK1, MAPK2, MAPK8, etc.), which has the function of regulating cell growth, differentiation, stress adaptation to the environment, inflammatory response, and other important cellular physiological and pathological processes [28]. Studies have also shown an unexpected mechanical link between MAPK signals and inflammatory network control during reprogramming caused by tumor therapy [29]. As can be seen from (Table 3), Cytokine Signaling in Immune system, Nanomaterial induced apoptosis, and PID HIV NEF PATHWAY may be Xiyanping injection anti-SARS-CoV-2 important biologic processes. In total, there are1599 GO biofunctions, of which 1447 are biological processes (BP), 61 are cell compositions (CC), and 91 are molecular functions (MF) (Figures 7(a), 7(b)). Most of the top 20 GO features are related to the reaction of response to an inorganic substance, cellular response to chemical stress, response to oxidative stress, and response to reactive oxygen species. We obtained 291 KEGG path enrichment features (Figures 8(a), 8(b)): 218 were related to infection and other diseases and 73 signaling pathways are mostly related to inflammation and immune pathways. Enriched by the DAVID platform [21] to 107 KEGG results, 47 correspond to a variety of diseases such as Hepatitis B, Chagas disease (American trypanosomiasis), colorectal cancer, and influenza A, tubeless. There are 60 pathways, the first three of which are TNF signaling pathways, the Toll-like receptor signaling pathway, and the HIF-1 signaling pathway, most of which are related to immune and inflammatory pathways, and we concluded that injection may be anti-SARS-CoV-2 through inflammation and immune pathways. Showing the TNF pathway (Figure 9), the sunflower represents Xiyanping injection, and the three arrows represent inhibition, dual-directional regulation, and active.

### 3.4. Analysis of Molecular Docking Results

It is generally believed that the smaller the binding energy of the ligand to the receptor, the greater the likelihood of its interaction and the easier the binding [30]. Andrographolide sulfonates include the following: Xiyanping injection, compound I, compound II, compound III, compound IV, and compound V; Yanhuning injection: VI and VII; Chuanhuning injection: VIII and IX. The degree value of the top 20 target proteins (Table 2) was selected for molecular docking with the above compounds. As can be seen from the molecular docking results, the binding energy of the target compound with the 20 target protein macromolecules is less than −5.0 k·J/mol [25]. Studies suggest that these ingredients may have anti-SARS-CoV-2 effects [2], and the results indicate that compounds III and Xiyanping injection have a good binding ability with target proteins. See heatmap for molecular docking binding energy (Figure 10). Colors range from red to blue. The bluer the color, the smaller the binding energy, the stronger the binding ability, and the better the docking results. Xiyanping injection and gene: HSP90AA1 (target protein: 3U93) has the highest Vina score of −9.7, Xiyanping injection, and HSP90AA1 (target protein: 3U93) docking mode (Figure 11).

The article "The Pharmacological Mechanism of Xiyanping Injection for the Treatment of Novel Coronavirus Pneumonia (COVID-19): Based on Network Pharmacology Strategy" was published in 2022. Journal: Evid Based Complement Alternat Med.

### 3.5. Organizing Enrichment Analysis

The differential expression of 93 gene targets in human tissue was analyzed using DAVID platform [21] Tissue Enrichment. As can be seen from (Figure 12), the redder the *P*-value circle, the greater the enrichment value, and the larger the count circle shape, the more enriched the gene. It can be seen that in tissues, placenta, liver, epithelial, lung, and other common target expressions are significant, of which the number of lung targets is 22. Among them, the results of molecular docking show that the high scores of Xiyanping injection Vina are HSP90AA1 and CAT gene target, and TNF and FOS gene target have higher compound III Vina scores. The expression of the above four genes in the respiratory and circulatory system was analyzed by the Human eFP Browser platform [26], and the distribution and absoluteness of the genes in the human body were analyzed (Figures 13–16). The higher the absolute, the redder the color, and the higher the gene expression. Human HSP90AA1 and other targets are believed to be effective potential therapeutics.

## 4. Discussion

According to the clinical trials of Zhang XY, Lv L, and Zhou YL, it can be proved that Xiyanping has the effect of treating COVID-19 [31]. Zhang XY, Lv L, Zhou YL, and others recruited 130 consecutive COVID-19 patients with mild-to-moderate symptoms from five research sites and randomly assigned them to receive Xiyanping injection combined with standard treatment or standard support treatment alone at a 1 : 1 ratio. The results showed that Xiyanping injection significantly reduced the time of cough relief, fever regression, and virus clearance. No serious adverse events were reported during the study. The above clinical trials can prove that Xiyanping has the effect of treating COVID-19, which is worthy of clinical promotion.

The article "The Pharmacological Mechanism of Xiyanping Injection for the Treatment of Novel Coronavirus Pneumonia (COVID-19): Based on Network Pharmacology Strategy" was published in 2022. Journal: Evid Based Complement Alternat Med.

The main component of Xiyanping injection is andrographolide, which is the main effective component of the natural plant *Andrographis paniculata*. It has the effects of dispelling heat and detoxification, anti-inflammatory, and analgesic. It has special effects on bacterial and viral upper respiratory tract infections and dysentery and is known as a natural antibiotic drug [32]. In clinical application of the product, its side effects are small. The median lethal dose of alcohol extracts of *Andrographis paniculata* in mice was 13.19 g/kg (calculated by andrographolide). The modern injection has adverse reactions because it directly enters the internal circulation without passing through the liver metabolism of the digestive system. The adverse reactions of andrographolide injections—Yanhuning injection and Chuanhuning injections—are more serious; therefore, they should be used with caution in children. China's National Medical Products Administration has reported security issues with Yanhuning injection/Chuanhuning injection and noted that Yanhuning injection/Chuanhuning injection was used cautiously for children [33]. In the consensus of experts on the clinical application of Xiyanping injection (Child Edition) in 2019, experts believed that Xiyanping injection can be used in children and has good clinical efficacy [1]. Xiyanping injection was recommended by multiple pediatric diseases guidelines/consensuses, and the adverse reactions were much smaller than those of similar drugs. In 2010, Xiyanping injection was recommended in the new editions of Hand, Foot and Mouth Disease Diagnosis and Treatment Guidelines, Influenza A (H1N1) Diagnosis and Treatment Programme, and Fever with Thrombocytopenia Prevention and Treatment Guidelines issued by the Ministry of Health (Table 4).

Excessive TNF can cause tissue damage, which is one of the core cytokines of an “inflammatory storm” caused by infection. TNF can induce cells to release cytokines, but in some cases, it can also induce apoptosis or programmed cell necrosis [34]. After Xiyanping injection enters the patient, its anti-inflammatory effect may be related to the TNF pathway, triggering many TNF pathway reactions: inhibiting TNFR1 and TNFR2 in the TNF pathway. At the same time, Xiyanping injection can regulate Caspase-3 and Caspase-8 in the Caspase family involved in the TNF pathway and mediate cell apoptosis. The activation of NFB JNK protein kinase-mediated by TRAF is inhibited by Xiyanping injection. Xiyanping injection inhibits the extracellular MAPK inflammatory pathway (inhibition of MAPK1, MAPK3, inhibition of MAP production), inhibits NF-*κ*B and other pathways in the nucleus through various pathways, inhibits the release of various inflammatory factors, and plays a role in the treatment of COVID-19.

The article "The Pharmacological Mechanism of Xiyanping Injection for the Treatment of Novel Coronavirus Pneumonia (COVID-19): Based on Network Pharmacology Strategy" was published in 2022. Journal: Evid Based Complement Alternat Med.

Target gene HSP90AA1: HSP90AA1 is an important regulator of inflammation because HSP90AA1 is currently understood as an extracellular agent secreted in wound healing and inflammation. Extracellular HSP90 + induces inflammation by activating NF-*κ*B (RELA) and STAT3 transcription procedures, including proinflammatory cytokines IL-6 and IL-8 [35]. In addition, it has an intracellular anticancer effect and induces autophagy. The anti-inflammatory mechanism of Xiyanping injection may be highly related to this target.

Target gene CAT: CAT gene occurs in almost all aerobic breathing organisms, which helps protect cells from the toxic effects of hydrogen peroxide. It promotes cell growth, including T cells, B cells, bone marrow leukemia cells, melanoma cells, breast cells, and normal and transformed fibroblasts [36]; Xiyanping injection may act on this target, anti-inflammatory effect.

Target gene TNF: TNF gene induces VEGF production by cooperating with IL1B and IL6 [37], plays an anti-inflammatory role, and plays a role in angiogenesis.

Target gene FOS: FOS is considered to play an important role in signal transduction, cell proliferation, and cell differentiation. In growth cells, phospholipid synthesis may be activated by CDS1 and PI4K2A [38]. This activity requires Tyr dephosphorization and association with the endoplasmic retina [38].

From the molecular docking Vina data, it was found that the overall score of compound III was better than that of Xiyanping injection. This also indicates the possibility of a potential new drug, with compound III having better water solubility than Xiyanping injection.

## 5. Conclusions

In this study, through network pharmacology, molecular docking, target analysis, and tissue analysis, it can be concluded that Xiyanping injection and andrographolide sulfonates such as compound III in the treatment of COVID-19 mainly act on HSP90AA1, CAT, TNF, FOS, and other targets. At the same time, Xiyanping injection inhibits the release of a variety of inflammatory factors by inhibiting intracellular MAPK, TNF, and other pathways and inhibiting NF-*κ*B and other pathways in the nucleus, thus playing a role in the treatment of COVID-19. Compound III is a potential new drug for the treatment of COVID-19. Xiyanping injection can achieve a therapeutic effect in patients with infectious pneumonia, which is in line with the “*Chinese Association of Traditional Chinese Medicine Expert Consensus* (literature reports)” [1] conclusion. In summary, Xiyanping injection is effective and safe in treating COVID-19, which is an important method for the treatment of COVID-19 in integrative medicine. The clinical practice and popularization and application are of far-reaching significance.

The article "The Pharmacological Mechanism of Xiyanping Injection for the Treatment of Novel Coronavirus Pneumonia (COVID-19): Based on Network Pharmacology Strategy" was published in 2022. Journal: Evid Based Complement Alternat Med.

## Figures and Tables

**Figure 1:** Technological roadmap of Xiyanping injection.

**Figure 2:** The structure of the compound.

**Figure 3:** 60 genes.

**Figure 4:** 93 genes.

**Figure 5:** The PPI networks for 89 genes.

**Figure 6:** The targets analysis.

**Figure 7:** (a) GO color by cluster; (b) GO color by *p*-value.

**Figure 8:** (a) KEGG color by cluster; (b) KEGG color by cluster.

**Figure 9:** TNF pathway.

**Figure 10:** Binding energy heatmap of some compounds with a target protein.

**Figure 11:** Xiyanping injection in combination with HSP90AA1.

**Figure 12:** Organizational enrichment differences.

**Figure 13:** Expression of HSP90AA1 in the human respiratory and circulatory system.

**Figure 14:** Expression of CAT in the human respiratory and circulatory system.

**Figure 15:** Expression of TNF in the human respiratory and circulatory system.

**Figure 16:** Expression of FOS in the human respiratory and circulatory system.

**Table 1:** 93 genes collected.

UniProt ID	Gene names
**P07900**	HSP90AA1
**Q9Y243**	AKT3
**P62937**	PPIA
**Q2M2I8**	AAK1
**Q9Y2I7**	PIKFYVE
**P31751**	AKT2
**P35613**	BSG
**Q99720**	SIGMAR1
**Q16774**	GUK1
**P27823**	PGA5
**P27824**	CANX
**P09651**	HNRNPA1
**P42684**	ABL2
**Q4KMQ2**	ANO6
**O15393**	TMPRSS2
**P09958**	FURIN
**P07711**	CTSL
**P01031**	C5
**P78536**	ADAM17
**P31749**	AKT1
**P51636**	CAV2
**P53779**	MAPK10
**P30530**	AXL
**Q9H2X3**	CLEC4M
**O76074**	PDE5A
**P68104**	EEF1A1
**Q02127**	DHODH
**P45983**	MAPK8
**P05121**	SERPINE1
**P06400**	RB1
**P26447**	S100A4
P48506	GCLC
Q16236	NFE2L2
P40763	STAT3
P08670	VIM
P04040	CAT
P12830	CDH1
Q15910	EZH2
P35968	KDR
P28482	MAPK1
P27361	MAPK3
P04637	TP53
P15336	ATF2
P10415	BCL2
P11802	CDK4
P10145	CXCL8
P20711	DDC
P49327	FASN
P00441	SOD1
P01375	TNF
P13500	CCL2
P29279	CCN2
Q9NSE2	CISH
P19875	CXCL2
P11712	CYP2C9
P08684	CYP3A4
P08246	ELANE
P17948	FLT1
P02751	FN1
P01100	FOS
P24298	GPT
P08721	SPP1
P15692	VEGFA
P05231	IL6
P42574	CASP3
P09601	HMOX1
Q14790	CASP8
P55957	BID
P05177	CYP1A2
P25445	FAS
P48023	FASLG
P05305	EDN1
P08253	MMP2
P14780	MMP9
P05164	MPO
P16284	PECAM1
P37231	PPARG
P04049	RAF1
P59594	ACE2
Q16665	HIF1A
P01137	TGFB1
Q14145	KEAP1
P13647	KRT5
O14733	MAP2K7
P45984	MAPK9
P01024	C3
P60842	EIF4A1
P00390	GSR
P00738	HP
P05412	JUN
P49841	GSK3B
P01033	TIMP1
P19320	VCAM1

**Table 2:** The top 20 genes for the degree value.

PDB ID	Target gene	Degree	UniProt ID	Protein name
6CCY	AKT1	75	P31749	RAC-alpha serine/threonine-protein kinase
4KVP	TP53	65	P04637	Cellular tumor antigen p53
4TWT	TNF	64	P01375	Tumor necrosis factor
4ZS7	IL6	62	P05231	Interleukin-6
6CKZ	CASP3	61	P42574	Caspase-3
6D3O	VEGFA	59	P15692	Vascular endothelial growth factor A
6QHD	STAT3	58	P40763	Signal transducer and activator of transcription 3
6MFA	JUN	57	P05412	Transcription factor AP-1
5J6Z	FN1	55	P02751	Fibronectin
2OW1	MMP9	54	P14780	Matrix metalloproteinase-9
6GES	MAPK3	51	P27361	Mitogen-activated protein kinase 3
4H6J	HIF1A	51	Q16665	Hypoxia-inducible factor 1-alpha
2O72	CDH1	49	P12830	Cadherin-1
2VV1	PPARG	49	P37231	Peroxisome proliferator-activated receptor gamma
4U93	HSP90AA1	47	P07900	Heat shock protein HSP 90-alpha
3IFD	CCL2	46	P13500	C-C motif chemokine 2
5D14	CXCL8	46	P10145	Interleukin-8
1CK7	MMP2	44	P08253	72 kDa type IV collagenase
7P8W	CAT	43	P04040	Catalase
1FOS	FOS	41	P01100	FOS G0S7

The article "The Pharmacological Mechanism of Xiyanping Injection for the Treatment of Novel Coronavirus Pneumonia (COVID-19): Based on Network Pharmacology Strategy" was published in 2022. Journal: Evid Based Complement Alternat Med.

**Table 3:** Network and annotation.

Network	Annotation
MyList	hsa05161|Hepatitis B|−41.7; R-HSA-1280215|Cytokine Signaling in Immune system|−39.3; ko04933|AGE-RAGE signaling pathway in diabetic complications|−38.8
MyList_MCODE_ALL	hsa05161|Hepatitis B|−47.8; hsa05200|Pathways in cancer |−46.3; WP4666|Hepatitis B infection|−42.3
MyList_SUB1_MCODE_1	hsa05161|Hepatitis B|−22.8; hsa05200|Pathways in cancer |−20.8; ko04933|AGE-RAGE signaling pathway in diabetic complications|−20.5
MyList_SUB1_MCODE_2	hsa05200|Pathways in cancer|−24.0; hsa05161|Hepatitis B|−23.3; ko05212|Pancreatic cancer|−22.9
MyList_SUB1_MCODE_3	R-HSA-194315|Signaling by Rho GTPases|−3.5; R-HSA-1280215|Cytokine Signaling in Immune system|−3.5; R-HSA-9716542|Signaling by Rho GTPases, Miro GTPases, and RHOBTB3|−3.5
MyList_SUB1_MCODE_4	R-HSA-1280215|Cytokine Signaling in Immune system|−4.2
MyList_SUB1_MCODE_5	WP384|Apoptosis modulation by HSP70|−9.6; WP2507|Nanomaterial induced apoptosis|−9.5; M197|PID HIV NEF PATHWAY|−8.8

**Table 4:** Xiyanping injection has been included in the guide/expert consensus list.

Serial number	Guideline/expert consensus name	Release year	Guidelines/expert consensus/formulation bodies
**1**	Hand-foot-mouth disease diagnosis and treatment guidelines (2010 edition)	**2010**	National Health Commission of the People's Republic of China
**2**	Guidelines for the diagnosis and treatment of viral pneumonia in children in TCM	**2011**	World Federation of Chinese Medicine societies
**3**	Expert consensus on integrated traditional Chinese and Western medicine treatment of acute fever in children	**2011**	Ma Rong, Wang Xuefeng, etc.
**4**	Guideline for clinical diagnosis and treatment of pediatrics of traditional Chinese medicine hand-foot-mouth disease (revised)	**2016**	China Association of Chinese Medicine
**5**	Clinical Diagnosis and Treatment Guidelines for Pediatrics of Traditional Chinese Medicine · Varicella (Revised)	**2016**	China Association of Chinese Medicine
**6**	Chinese medicine pediatric clinical diagnosis and treatment guidelines bacillary dysentery (formulation)	**2017**	China association of Chinese medicine
**7**	Expert Consensus on Diagnosis and Treatment of Mycoplasma Pneumoniae Pneumonia in Children by Integrated Traditional Chinese and Western Medicine (2017)	**2017**	China Association of Chinese Medicine of Pediatric Pneumonia Alliance
**8**	Expert Consensus on Clinical Application of Xiyanping Injection (for Children)	**2019**	Institute of Basic Research In Clinical Medicine/China Academy Of Chinese Medical Sciences
**9**	The new diagnosis and treatment scheme for coronavirus pneumonia (trial version 4)	**2020**	National Health Commission of the People's Republic of China / National Administration of Traditional Chinese Medicine
**10**	The new diagnosis and treatment scheme for coronavirus pneumonia (trial version 5)	**2020**	National Health Commission of the People's Republic of China/National Administration of Traditional Chinese Medicine
**11**	The new diagnosis and treatment scheme for coronavirus pneumonia (trial version 6)	**2020**	National Health Commission of the People's Republic of China/National Administration of Traditional Chinese Medicine
**12**	The diagnosis and treatment scheme of new coronavirus pneumonia (trial version 7)	**2020**	National Health Commission of the People's Republic of China/National Administration of Traditional Chinese Medicine
**13**	New coronavirus pneumonia diagnosis and treatment plan (trial version 8)	**2020**	National Health Commission of the People's Republic of China/National Administration of Traditional Chinese Medicine

The article "The Pharmacological Mechanism of Xiyanping Injection for the Treatment of Novel Coronavirus Pneumonia (COVID-19): Based on Network Pharmacology Strategy" was published in 2022. Journal: Evid Based Complement Alternat Med.

## Data Availability

All data used to support the findings of the study are included within the article.
